This article has been retracted.

# Analysis and Application of Language Environment Function from the Perspective of English Linguistics

**DOI:** 10.1155/2022/1757002

**Published:** 2022-07-08

**Authors:** Lin Zhu

**Affiliations:** ^1^School of Foreign Study, Henan Polytechnic University, Jiaozuo 454000, China; ^2^Department of English, Chosun University, Gwangju 501759, Republic of Korea

## Abstract

In recent years, more and more questions have been raised about the idea that a sentence alone can fully analyze the semantics without considering the context. When we talk about the acceptability of a sentence, we immediately and naturally think of the context in which the sentence can be used correctly. In the current English classroom teaching, teachers follow the traditional teaching procedures too much: first give detailed explanations, and then carry out mechanical exercises. The lack of flexible teaching methods and the creation of contexts affects the improvement of students' communicative ability. During my long-term learning of English, I have considered the following questions: how to make use of the function of context to make English learning diverse and challenging; how to create a variety of practical forms, such as creating a way to make students interested and able to participate in learning, in order to improve students' language communication ability. This paper analyzes the current situation of English teaching, expounds the concept and classification of context and language application, summarizes the applied linguistics theory and related theory, and analyzes the context of English linguistics horizon function and application. This study combines context with English learning, and English learning “how to create and use context,” so as to improve students' communicative competence.

## 1. Introduction

The 21st century is an era of great economic development. With the continuous advancement of global integration, China has become more open to the world, and English is used more and more frequently in China. And with the development of economic globalization, all walks of life have a relatively large demand for English-related talents, and at the same time, it also provides a good learning environment for talent training. In recent years, cultural exchanges between my country and other countries have become more and more frequent, and the opportunities for communication in the English context have gradually increased. English linguistics is a kind of language education. Only through practical communication can the ability be truly improved.  Table 1 shows the ranking of English proficiency in countries around the world. As can be seen from the table, the proficiency of English in all regions of China is only medium, which has a lot to do with the language environment we live in. The development of economy provides a language environment for personnel training, which can cultivate students' speaking ability, listening ability, etc., which is beneficial to the development of English linguistics.

As a world language, more and more people are aware of the importance of learning English.  Figure 1 shows the market size and growth rate of my country's English training industry. According to the figure, China's English literacy training industry reached its peak in 2021 and its lowest point in 2020, which is mainly affected by the epidemic. In the process of learning English, one is exposed to the English context, can get a better learning effect, and create a strong English context through interactive methods and communication platforms, making language learners immersive. Language is an important carrier and basic content for people to communicate and communicate. Only by paying attention to the connection between context and semantics from the perspective of linguistics can we achieve better and more accurate understanding of English content. Because the context helps the learners to judge the semantics, this makes the semantics single and concrete. In order to create a strong English learning atmosphere, learners need to learn English in connection with the English context in their daily life. In general, context plays a driving role in integrating learning in English linguistics and mastering English language knowledge. Based on this situation, it is of great practical significance to explore the integration and practical application of context in the English language perspective.

## 2. Theoretical Research

### 2.1. Overview of English Linguistics

Whether it is a modern language or an ancient language, it is an objectively existing language phenomenon [1]. Although the meanings expressed by different discourses are subjective and varied, linguistics can be defined as “the discipline of learning language,” a definition widely accepted because it succinctly points out that linguistics is the goals and methods of a discipline [2]. The object of linguistics is language, and it studies all languages [3]. Linguistics includes functional linguistics (pragmatics), cognitive linguistics, applied linguistics (foreign language teaching), translation, etc. In linguistics, English linguistics is an important branch.

English linguistics is a basic compulsory course in English learning, and its importance is self-evident. The goals of the course include systematically imparting knowledge of modern linguistics, improving students' English learning ability, stimulating students' interest in language research, and cultivating students' innovative ability [4]. In the study of English linguistics, it is necessary to focus on understanding the culture of English-speaking countries, to ensure that it conforms to the rules and regulations of English language application in actual use, and to achieve barrier-free communication with people. In actual teaching, it is necessary to construct a suitable context, so as to achieve the effect of improving students' English learning and comprehension level and English application and practice ability [5]. At the same time, English linguistics is an important part of learning English. Even in English-speaking countries, English linguistics requires students to study hard. The so-called language is that in the long-term accumulation process of life, people summarize the pronunciation into fixed syllables and pronounce according to a certain structure and sequence and then express their wishes. English linguistics reflects the living environment of English-speaking countries, including cultural background, way of thinking and old habits [6]. If you want to use them accurately, you must abide by these rules to achieve the purpose of communicating with people.  Figure 2 shows the mastery of English in Asian countries [7]. As can be seen from the picture, among the Asian countries, only Singapore has a high English level, and there are still some problems in English communication in China.

### 2.2. Context

#### 2.2.1. What Is Context

Context is the environment where the language is used. Internal context refers to the relationship between a certain speech segment and a certain context, and external context refers to the social environment of the language existing outside of the speech fragment. Linguists put forward the hope to determine the correctness of language use in the process of determining the usage of sentence patterns, that is, to consider the accuracy of language use on the basis of context. The Polish human linguist Malinowski believes: “Discourse and environment are closely intertwined, and language environment is essential for understanding language” [8]. Any linguistic analysis involving context will belong to the field of linguistics research. The definition of context in linguistics: the language environment refers to the situation and state in which a person is speaking [9]. Generally speaking, the natural context is the living environment in which the language is the mother tongue; the local context is the learner's part-time living or learning in the language environment; and artificial language context is a language in which the learner retells, describes, memorizes, or creates certain scenes in their minds [10].

Language is a social phenomenon and a social activity. Therefore, the use of language is always inseparable from a certain context, just like the growth of plants is inseparable from soil and water. Therefore, when learning English language, not only must we try our best to understand the language knowledge, such as pronunciation, vocabulary, and grammar, but also be good at understanding the meaning of language accurately in a certain context and improve the ability to use the English language in practice [11].

#### 2.2.2. The Role of Context

When language analysts conduct language research, they will inevitably choose a pragmatic approach to consider language issues [12]. It is difficult to accurately understand the semantics of words, and they do not understand the grammar of sentences, so that scholars cannot master good English learning methods. That is, language analysis must be combined with the background of utterance. The role of context includes the following: The first is the reference function. It means that in the process of studying linguistics, linguists can judge the meaning of a word according to the context, which is more conducive to accurately expressing the meaning of the word. Combined with the context, it has a certain reference for the understanding of the meaning of the word, helping learners to better understand the meaning of words; good grasp of vocabulary meaning.

The second is supplementary effect [13]. The supplementary effect of English context on language understanding is mainly reflected in the understanding of the deep meaning and implication of the language. A sentence may express not only the simple literal meaning but also a deep meaning given by the context. It may be an implication beyond the literal meaning. The literal meaning is easier to understand, but it is not so easy to understand the meaning of each word and the complete meaning of the combination of words in the context [14].

The third is restrictive effect. The restrictive effect of context on language use is first manifested in the understanding and selection of words. The meaning of the same word in different contexts may be different. At this time, an accurate understanding should be made according to the specific context. To understand the meaning of a word correctly requires analysis in combination with the actual context. Secondly, the limiting effect of context on language use is reflected in the understanding and organization of sentences. It is easier to understand when the completed sentences are connected together. If they are separated, it will make people feel confused [15]. Finally, the limitation of context on language use is also reflected in the understanding and arrangement of paragraphs and the whole article. If readers suddenly read an article about American dining rules, they must not be able to understand their dining culture, but if they are familiar with the foundations of American dining culture. After reading the related articles, it will be easier to understand the meaning of the scenes described in the text [16].

#### 2.2.3. Categories of Context

The English context category includes situational context. British linguist Lyons will interpret the context as abstracted from the actual situation and some factors that affect speech activities, involving both parties, occasions, and speaking. In the natural context, verbal communication is always carried out in a certain time and space, and verbal expression will be affected by seasonal, geographical environment, natural scenery, and other factors. In the appropriate natural context, the language organization and expression can arouse the resonance of the other party and achieve a better expression effect; in the cultural context, the expression of some words can only play their real role if they are expressed in a specific cultural context [17]. Under the influence of different backgrounds such as history, culture, customs, values, and living habits, specific language expressions will produce different language effects. Cognitive context involves three types of language knowledge application categories: situational knowledge, language context, and cognitive background knowledge. According to the needs of different occasions, language users will consciously or unconsciously activate the content of the serious context, making the dialogue between people more in line with etiquette [18].

## 3. Functional Analysis of Context from the Perspective of English Linguistics

Adding context in the process of learning English has two effects on students' English learning: first, it helps to quickly understand new words. Vocabulary is the basic content of learning a country's culture and language. Combined with the development of thinking training based on different contexts, it can promote learning individuals to deeply integrate into the corresponding country's culture. In the process of learning new words, in addition to understanding their fixed meanings, they should also be integrated into specific situations to understand and master the different semantics of new words; and second, it helps to eliminate misunderstandings [19]. In the process of English application, there are common misunderstandings, for example, memorizing words by rote and cannot be flexible, and these misunderstandings generally originate from differences in thought, national culture, and other aspects. Relying on the integration of context in English learning, it can achieve the effect of eliminating these misunderstandings and promote the learning individual to truly understand the meaning of the sentence [20].

### 3.1. Judging Polysemy of Words

There are many words in English that have the same meaning as Chinese. For example, a word will have different meanings, and different meanings of the word will have different meanings when used in different contexts, so learners must be able to clearly understand the context in which the word is used in the sentence and its true meaning. Through the analysis and research of English context, learners can truly understand the context in which the word is used and finally judge the meaning of the word. Since the expression and meaning of a word in different contexts are quite different, only by reasonably grasping and understanding the context in which English words are used can the whole text be better penetrated and smooth communication between learners can be facilitated. In the process of English language research, scholars will find that English words and Chinese word research have similarities. The same words will express different meanings, and how to correctly understand the meaning of words has become a problem that researchers need to think about. Learn from Chinese research based on our experience, we can apply the context function to linguistic research to judge the multiple meanings of English words through context. When conducting English language research, only by figuring out the multilayered meaning of each word and the grammar of the paragraph can we better understand the meaning of the whole sentence. The context of an English word is different, and the meaning expressed is completely different. If you want to judge the meaning of an English word in a sentence, you must first contact its context, that is to say, the context has the function of helping readers to judge English polysemous words.  Figure 3 shows the basic grammar knowledge in English learning. Only by understanding the grammar knowledge and learning to integrate the context can you improve your English level.

### 3.2. Understanding English Texts

When linguists analyze the meaning of a sentence, in addition to carefully translating each word and figuring out the grammar used in each sentence, they also need to understand the context of the entire sentence and even the paragraph because the meaning of each word and sentence may be different. Only by placing it in a certain context can we accurately grasp the meaning of words and sentences, and when we conduct language research, we can understand the thoughts and emotions conveyed by the article. For example, when you see the sentence “I want breaking up with you”, you will think that the two people who are talking are lovers. In fact, using this sentence on different occasions can also express the relationship between good friends' emotion. Many times when we understand the meaning of a sentence, we will be ambiguous. It is because we have not really entered the context of the sentence, which will lead to deviations in understanding, so the context helps to understand the entire English text—the meaning of the article. Only understanding English chapters can help improve students' reading ability.  Table 2 shows the English reading ability of Chinese and American students. It can be seen from the table that Chinese students' English reading ability is 2–3 levels lower than that of American students.

### 3.3. Understand English Vocabulary Related to Cultural Background

In the process of continuous development, human beings have produced a variety of cultural types, and each country, each nation, and different regions will have differences in culture, which also makes it difficult for us to learn English and use context. With the help of contextual learning, learners can deepen their understanding of the vocabulary. Learners should also master the cultural backgrounds of different countries, which will facilitate the communication of learners in different environments. After understanding the basic background, they can roughly understand its meaning. The mastery of contextual grammar is inextricably linked with the cultures of different countries. When learning the context, contacting the cultures of various countries can deepen learning and memory. When we cannot fully understand the customs and culture of a place, how can we avoid the embarrassing situation caused by the wrong use of semantics? Then, it is a good way to understand the meaning of words according to the context. To understand the meaning of people's words with the help of context, maybe we can only roughly understand the meaning of other people's expressions, but with the help of context, we can make our communication process smoother. Once upon a time when the great British writer Dickens went to the United States on a business trip and stayed in a hotel, the waiter asked him, “Would you like have your dinner right away?” “right away” means “immediately, right away” in American English, so the waiter meant to ask Dickens if he wanted dinner now, and Dickens thought the waiter was asking him if he needed to go outside Meal; this is the misunderstanding caused by differences in understanding of English vocabulary under different cultural backgrounds.

### 3.4. Improve Speaking Ability

Oral ability is the most important item in English ability. Only by mastering oral ability can we communicate with others normally; for example, students' ability to hear, read, and write when learning English. Through oral practice, other abilities can be improved at the same time. Judging from the current situation of English language learning, young people in our country are generally weak in spoken English, and many students have learned English but dare not communicate in language. And without oral communication, English learning is incomplete and difficult to apply in the future. Many people will have poor oral English when learning English, especially young people in my country, who are reluctant to open their mouths to express themselves when learning English, so they cannot really improve their oral English ability. With the development of internationalization, English communication has become a very common phenomenon. Creating a good language environment is an effective way to help people improve the level of oral communication. In this context, people do not need to consider whether each other's pronunciation is very accurate but must exercise their own expression skills, correct their own pronunciation, and then continuously improve the level of oral expression. Therefore, students do not need to worry about nonstandard pronunciation. As long as they muster up the courage to practice continuously and make corrections in communication, they can gradually improve their speaking ability. In order to judge the English level of individuals, our country has developed the English level evaluation shown in Table 3—a scale through which one can know what their speaking level is.

### 3.5. Assimilate Surrounding People

Subtle influences on people's thoughts and characters will be subtly affected, and these influences come from the outside world. Learners who have been exposed to good influences for a long time will be nurtured. During this period, the students live a Chinese life. They can eat with chopsticks, wear Chinese clothes, and speak Chinese, sing Chinese songs. Under the influence of such a sinicized life, American teenagers have been subtly influenced, and their own Chinese listening and speaking ability has also been significantly improved.

## 4. The Application of Contextual Functions from the Perspective of English Linguistics

### 4.1. Applying Contextual Functions in Spoken Communication

In the process of oral communication, we should understand the background environment in which the language occurs, so as to choose the correct vocabulary and use methods to ensure the smoothness of communication. A mastery of context enables conversations to take place effectively, both as the narrator and as the listener. In the process of expressing language, the narrator must fully consider the background of the dialogue, the living environment, and social background of the listener and express on this basis, so as to ensure the accuracy of the words and sentences used, so that the listener can accurately understand. Therefore, the narrator should be able to correct errors according to the content of the context and modify the sentences according to the content of the article, so as to achieve efficient dialogue and communication.  Figure 4 shows the learning methods chosen by Chinese parents to improve oral communication skills for students of all ages. According to the picture, parents of children or cities are willing to send their children to English learning institutions for training.

### 4.2. Use Contextual Functions in Various Communications

Context is the premise of language communication, and a good language environment can drive learners' desire to communicate. According to the survey, in the face of a negative language environment or when the conversation cannot attract the attention of the other party, the learners' language expression is not accurate. On the one hand, it is because the learners are in a tense state in this environment and cannot really express their language ability; obstacles or even reluctance to communicate. Therefore, language experts should create a good language communication environment for learners, so as to stimulate the desire of learners to communicate, and it is best to actively guide learners to communicate in the process of communication. Therefore, it is very important to establish a good language communication environment; through the context function can really achieve the effect of improving the English level of learners.

### 4.3. Applying Contextual Functions in a Networked Language Environment

The learning of any language includes the influence of personal ability and the driving of the external environment. In English linguistics, context function is the most important aspect that affects language learning ability. By creating context, it can help learners find their own learning methods, find problems in the context, and solve problems effectively. With the development of science and technology, the impact of the Internet on people's lives is getting bigger and bigger. The Internet platform has a great impact on language communication. Nowadays, the communication between people is not limited to face-to-face communication, and even most of them are inclined to the communication on the Internet platform. The establishment of the context is even more important under this kind of platform communication.  Figure 5 shows the growth rate of my country's youth population and the corresponding online English penetration rate. In face-to-face communication, the establishment of context is easier because the state of communication can be easily analyzed through the surrounding environment and body movements.

## 5. Conclusion

The development of the economy has made the English language more and more widely used, and it has also had a great impact on people's lives. In order to ensure the smooth progress of the communication, the most suitable communication method for both parties can be found through the analysis of the context. For different contexts, the communication methods used are different, and the sentences and vocabulary used are also different. This is a technique that needs to be carefully studied. By judging the sentences, we can better understand the article in depth, so as to understand the voice of the author or narrator. Not only that, through specialized research on context, learners can also improve their basic English knowledge and speaking ability.

To sum up, in the analysis and application of contextual functions in English linguistics, this paper first starts from the contextual research in English linguistics to clarify what context is, the role of context, and the categories of context, and then the context function in English linguistics is analyzed, including judging English polysemous words, understanding English texts, understanding English vocabulary related to cultural background, and improving speaking ability. Including the application of context functions in oral communication, in various exchanges and in the network language environment, through the above research, we hope that every linguist can realize the importance of context in language research.

## Figures and Tables

**Figure 1:** Market size and growth rate of China's English literacy training industry from 2017 to 2023.

**Figure 2:** Asian countries' English mastery level.

**Figure 3:** Basic English grammar framework.

**Figure 4:** Chinese parents' choices for improving oral language for children of different ages.

**Figure 5:** My country's youth population growth rate and online English penetration rate.

**Table 1:** Ranking of English proficiency indicators by countries in the world.

Very high proficiency	High proficiency	Medium proficiency	Low proficiency
1 Netherlands	15 Hungary	30 Costa Rica	47 Belarus
2 Sweden	16 Romania	31 France	48 Russia
3 Norway	17 Serbia	32 Latvia	49 Ukraine
4 Denmark	18 Kenya	33 Hong Kong, China	50 Albania
5 Singapore	19 Switzerland	34 India	51 Bolivia
6 South Africa	20 Philippines	35 Spain	52 Vietnam
7 Finland	21 Lithuania	36 Italy	53 Japan
8 Austria	22 Greece	37 South Korea	54 Pakistan
9 Luxembourg	23 Czech republic	38 Taiwan, China	55 Bahrain
10 Germany	24 Bulgaria	39 Ma Gugui	56 Georgia
11 Poland	25 Slovakia	40 China	57 Honduras
12 Portugal	26 Malaysia	41 Macau, China	58 Peru
13 Belgium	27 Argentina	42 Chile	59 Brazil
14 Croatia	28 Estonia	43 Cuba	60 El Salvador
	29 Nigeria	44 Dominican Republic	61 Indonesia
		45 Paraguay	62 Nicaragua
		46 Guatemala	63 Ethiopia
			64 Panama
			65 Tunisia
			66 Nepal
			67 Mexico
			68 Colombia
			69 Iran

**Table 2:** Comparison of English reading ability of Chinese and American students.

American education grade	U.S. education level	Lexile level	Chinese education grade
American preschool		0L to 100L	Chinese preschool
American preschool		100L to 200L	Chinese primary school grades 1–3
American preschool		150L to 300L	Chinese primary school grades 4–6
1st grade American elementary school	1st grade	200L to 400L	Chinese junior high school grade 1
2nd grade American elementary school	2nd grade	300L to 500L	Chinese junior high school grade 2
3rd grade American elementary school	3rd grade	500L to 700L	Chinese junior high school grade 3
4th grade American elementary school	4th grade	650L to 850L	Chinese high school grade 1
5th grade American elementary school	5th grade	750L to 950L	Chinese high school grade 2/3
6tht grade American elementary school	6th grade	850L to 1050L	Year 1 of Chinese university
American junior high school grade 1	7th grade	950L to 1075L	Year 2 of Chinese university
American junior high school grade 2	8th grade	1000L to 1100L	Year 3 of Chinese university
American junior high school grade 3	9th grade	1050L to 1150L	Year 4 of Chinese university
American high school grade 1	10th grade	1100L to 1200L	1st year postgraduate students in China
American high school grade 2/3	11th and 12th grade	1100L to 1300L	2nd year postgraduate students in China
SAT, GRE, GMAT, CAST		1300L	Chinese doctoral students

**Table 3:** Chinese English proficiency evaluation scale.

Scale registration		Roughly corresponds to the learning stage		National English Proficiency Test	
High	9	High-end foreign language talents		Level 9 (redevelopment on demand)	
	8			Level 8 (redevelopment on demand)	
	7	English major		Level 7	
Low	6	University	So hard		Level 6
	5		Basic requirements		Level 5
	4	High school		Level 4	
	3	Junior high school		Level 3	
	2	Primary school		Level 2 (evaluation only)	
	1			Level 1 (evaluation only)	

## Data Availability

The labeled data set used to support the findings of this study is available from the corresponding author upon request.
